The article "Effect of metals on the regulation of acidogenic metabolism enhancing biohydrogen and carboxylic acids production from brewery spent grains: Microbial dynamics and biochemical analysis" was published in 2022. Journal: Eng Life Sci.

# Effect of metals on the regulation of acidogenic metabolism enhancing biohydrogen and carboxylic acids production from brewery spent grains: Microbial dynamics and biochemical analysis

**DOI:** 10.1002/elsc.202200030

**Published:** 2022-08-30

**Authors:** Omprakash Sarkar, Ulrika Rova, Paul Christakopoulos, Leonidas Matsakas

**Affiliations:** ^1^ Biochemical Process Engineering Division of Chemical Engineering Department of Civil, Environmental, and Natural Resources Engineering Luleå University of Technology Luleå Sweden

**Keywords:** acidogenesis, biohydrogen, carboxylic acids, caproic acid, carboxylic acids, caproic acid metals

## Abstract

The present study reports the mixed culture acidogenic production of biohydrogen and carboxylic acids (CA) from brewery spent grains (BSG) in the presence of high concentrations of cobalt, iron, nickel, and zinc. The metals enhanced biohydrogen output by 2.39 times along with CA biosynthesis by 1.73 times. Cobalt and iron promoted the acetate and butyrate pathways, leading to the accumulation of 5.14 gCOD/L of acetic and 11.36 gCOD/L of butyric acid. The production of solvents (ethanol + butanol) was higher with zinc (4.68 gCOD/L) and cobalt (4.45 gCOD/L). A combination of all four metals further enhanced CA accumulation to 42.98 gCOD/L, thus surpassing the benefits accrued from supplementation with individual metals. Additionally, 0.36 and 0.31 mol green ammonium were obtained from protein‐rich brewery spent grain upon supplementation with iron and cobalt, respectively. Metagenomic analysis revealed the high relative abundance of *Firmicutes* (>90%), of which 85.02% were *Clostridium*, in mixed metal‐containing reactors. Finally, a significant correlation of dehydrogenase activity with CA and biohydrogen evolution was observed upon metal addition.

## 1 INTRODUCTION

Conversion of biomass to fuels and chemicals has become a priority owing to the increasing cost, progressive depletion, and greenhouse gas emissions associated with fossil‐based feedstock. Biomass‐derived fuels and chemicals could prevent the emission of 466 million tons of greenhouse gases by 2030, highlighting their potential environmental and economic benefits [1]. Acidogenic (dark) fermentation represents an intermediate stage of anaerobic digestion, offering an attractive and environmentally friendly way of converting biomass to renewable fuel and chemicals, such as biohydrogen and short‐chain or medium‐chain carboxylic acids (SCCA and MCCA, respectively) [2, 3, 4, 5]. However, the yield and efficiency of the acidogenic fermentation process depends on many factors, such as nature of the biocatalyst, redox conditions, substrate type, and presence of metals [6]. An optimal concentration of metals, including iron, cobalt, nickel, zinc, copper, and magnesium, in the reactor can significantly enhance the output of metabolites [2, 7, 8]. Metals are intimately involved in numerous life processes [9]. Metals have a specific function within the metabolic pathways of anaerobic microorganisms, thus affecting H_2_ and CA production [3, 10] (Table 1). Nickel and iron constitute the active site of [Ni–Fe] and [Fe] hydrogenases, which catalyze the reduction of protons to H_2_. In addition, iron is essential for the formation of ferredoxin, whose [Fe–S] center acts as an electron carrier during the oxidation of pyruvate to acetyl‐CoA and CO_2_. Addition of nickel increases bioH_2_ production. Cobalt is an ingredient of the corrin ring of coenzyme B_12_(cyanocobalamin)‐containing enzymes, which are important for bioH_2_ generation during microbial fermentation [2, 11].

The article "Effect of metals on the regulation of acidogenic metabolism enhancing biohydrogen and carboxylic acids production from brewery spent grains: Microbial dynamics and biochemical analysis" was published in 2022. Journal: Eng Life Sci.

**TABLE 1:** Influence of various metals addition on acidogenic fermentation

**Substrate**	**Metal concentration (mg/L)**	**Biohydrogen**	**References**
Potato waste	Fe^2+^ (0–1000)	4.98 L	[44]
Potato waste	Ni^2+^ (500)	0.18 L	[44]
Sucrose	Fe^2+^ (0–3200)	0.35 L	[45]
Glucose	Zn^2+^ (0–500)	1.73 mol/mol glucose	[46]
Wastewater	Ni nanoparticles (20–100)	0.024 L/gCOD	[47]
Activated sludge	Ni^2+^ (0–500)	0.1–80 ml/mgCOD	[48]
Glucose	Co‐Fe nanoparticles (100–500)	0.21L/g glucose	[49]
Wastewater	Ni^2+^ (0–64)	14.89 mol kg/COD_R_	[30]

Crucially, when the concentration of the added metals or elements is outside the optimal range, the acidogenic process is slowed or hampered (particularly with single culture). Most studies have focused on enhancing production of acidogenic metabolites by supplementing the required metals within the optimum range. However, the influence of elevated concentrations of metals on acidogenic fermentation remains mostly unexplored for mixed culture. The metal concentration in this investigation was chosen based on existing literature. Further, the study describes the effect of high amounts of metals on acidogenic fermentation, with the aim of selecting for microorganisms capable of withstanding a metal shock. A metal‐rich environment was previously shown to lead to the development of plasmid‐borne resistance systems in microorganisms, particularly among Eubacteria [9]. To identify the most relevant microorganisms in a high‐metal environment, metagenomics analysis was conducted during the biosynthesis of CA and bioH_2_ from brewery spent grains (BSG) as substrate. As, only a little is known on the dynamics of microbial populations that inhabit high concentration of a particular metal in the reactor. This study is also important towards development of selectively enriched biocatalyst using metals. Developing a biocatalyst that regulates the process, in particular to produce biobased chemicals and fuels from waste streams is not a straightforward, task. It has only been made possible by using a variety of preparation methods, (physical and chemical methods) each of which is quite expensive [12, 13, 14]. This approach provides an avenue to understand the influence of metals on acidogenic fermentation and to regulate the process by developing an effective consortium transforming biomass to chemicals and fuels.

The article "Effect of metals on the regulation of acidogenic metabolism enhancing biohydrogen and carboxylic acids production from brewery spent grains: Microbial dynamics and biochemical analysis" was published in 2022. Journal: Eng Life Sci.

**PRACTICAL APPLICATION**

Metals/elements are intimately involved in numerous life processes having a specific function within the metabolic pathways in microbes, affecting their metabolites formation. Metals/elements can significantly enhance the acidogenic metabolites such as carboxylic acids and biohydrogen. This study is important for developing an enriched acidogenic biocatalyst using metals/elements. As the development of a biocatalyst to regulate the process for an enhanced production of biobased chemicals and fuels from biomass is not a straightforward task, which has only been possible by employing different pretreatment methods. This approach provides an avenue to regulate the process by developing an effective consortium transforming biomass into chemicals and fuels.

## 2 MATERIAL AND METHODS

### 2.1 Biocatalyst and feedstock

Anaerobic sludge used as microbial culture was collected from the Luleå biogas plant, Luleå, Sweden. Before use, the sludge was filtered using a stainless‐steel mesh to remove any grit and other solid particles (e.g., hair and paper), and allowed to settle overnight. Following removal of the supernatant (mostly water), the thickened sludge presented a volatile solids (VS) content of 0.26 g/g. To promote an active bacterial population, the sludge was incubated at ambient temperature for 72 h with a nutrient solution containing 3 g/L glucose. No other micro or macronutrient were added during the incubation period. BSG used in this study was provided by Skellefteå Bryggeri (Skellefteå, Sweden). The homogenized BSG consisted of 96.2% ± 0.02% w/w total solids, of which 94.2 ± 0.03% w/w were VS. Cellulose, hemicellulose, and lignin accounted for 29.35%, 16.64%, and 13.33% w/w of BSG, respectively. Further, the BSG's amino acid composition was analyzed and found with its value of 17.97 g/100 g BSG.

### 2.2 Experimental design

The experiments were conducted in 18 identical 2 L glass bottle reactors (triplicates of six experiments) using the AMPTS‐II analyzer (Bioprocess Control, Lund, Sweden). The reactors were equipped with a motor to allow for mixing. All reactors were inoculated with cultures (10% v/v), fed with BSG (70 gVS), and filled with up to 1.2 L tap water. Four reactors were supplemented with cobalt (700 mg/L CoCl_2_), iron (7000 mg/L FeCl_2_), nickel (600 mg/L NiCl_2_), and zinc (800 mg/L ZnCl_2_). A fifth reactor served as control (no metals added), and a sixth reactor contained a combination of all four metals to evaluate their synergistic effect. Each reactor has a unique code on its label (Table 2). No additional nutrients/elements were added, as BSG itself was sufficiently rich. Prior to start up, the pH of the fermentation media was adjusted to 7.0 using 2 M HCl/NaOH. To establish anaerobic conditions, N_2_ gas was sparged into the reactor for about 30 minutes. For 72 days, all reactors were run in batch mode under mesophilic conditions (35°C). The average results and standard deviation were provided for all fermentation tests and measurements, which were carried out in triplicate.

The article "Effect of metals on the regulation of acidogenic metabolism enhancing biohydrogen and carboxylic acids production from brewery spent grains: Microbial dynamics and biochemical analysis" was published in 2022. Journal: Eng Life Sci.

**TABLE 2:** Reactors containing individual, or combinations of metals supplemented during acidogenic fermentation of BSG at a defined organic load

Metal	Reactor	Concentration (mg/L)	Metal (mg/gVS_load_)	Fermentation time (days)
Cobalt	R_Co_	700	10	72
Iron	R_Fe_	7000	100	72
Nickel	R_Ni_	600	8.57	72
Zinc	R_Zn_	800	11.43	72
Control	R_CTRL_	0	–	72
Mixture (cobalt+iron+nickel+zinc)	R_MIX_	700 + 7000 + 600 + 800	130	72

### 2.3 Analytical methods

The process parameters during fermentation were assessed by monitoring tchemical oxygen demand (COD) with respect to total CA output, redox conditions, dehydrogenase activity, biogas generation, and microbial population. Alcohol and carboxylic acid content was analyzed using a high‐performance liquid chromatography system (PerkinElmer, Waltham, MA, USA) equipped with a 410 LC pump and RID‐6A refractive index detector (PerkinElmer). The Aminex HPX‐87H column (300 m × 7.8 mm; Bio‐Rad, Hercules, CA, USA) was maintained at 65°C. The mobile phase consisted of 5 mM H_2_SO_4_, which was eluted at 0.6 ml/min. The biogas collected in the gasbag connected to the headspace of the reactor was analyzed using a mass spectrometer (GAM 400; InProcess Instruments, Bremen, Germany). SCCA and MCCA were quantified using calibration curves generated from commercially available standards (10 mM, volatile free acid mix; Sigma‐Aldrich, St. Louis, MO, USA). Dehydrogenase activity was estimated by a colorimetric procedure based on the reduction of 2,3,5‐triphenyltetrazolium chloride (TTC) [15].

### 2.4 DNA extraction, library preparation, and processing of DNA sequencing

To evaluate microbial diversity, samples were collected from the reactors on day 72. DNA was extracted using the FastDNA Spin Kit for Soil (MP Biomedicals, Santa Ana, CA, USA). Briefly, 500 μl of sample was transferred to a lysis matrix tube, followed by addition of 480 μl sodium phosphate buffer and 120 μl MT buffer. Bacterial cells were broken by bead beating at 6 m/s for 4 × 40 s. A TapeStation 2200 electrophoresis unit and Genomic DNA ScreenTape (Agilent Technologies, Santa Clara, CA, USA) were used to validate size and purity of a subset of DNA extracts. DNA was quantified with the Qubit dsDNA HS/BR Assay (Thermo Fisher Scientific, Waltham, MA, USA). Finally, 10 ng of extracted DNA was used as template for PCR amplification, together with 12.5 μl PCRBIO Ultra Mix (PCRBiosystems, Oxford, UK) and forward and reverse tailed primers (400 μM). The tailed primers were prepared by adapting an Illumina protocol [16] and contained sequences targeting the bacteria/archaea 16S rRNA gene variable region 4(abV4‐C): GTGYCAGCMGCCGCGGTAA (515FB) and GGACTACNVGGGTWTCTAAT (806RB). Taxonomy was assigned using the uclust classifier implemented in the assign_taxonomy.py script in QIIME and the MiDAS database, release 481 [17]. All bioinformatic processing was done in RStudio IDE (1.4.1717) running R version 4.1.0 (2021‐05‐18) and using R packages ampvis (2.7.8), tidyverse (1.3.1), seqinr (4.2.8), ShortRead (1.50.0), and iNEXT (2.0.20) [18, 19].

The article "Effect of metals on the regulation of acidogenic metabolism enhancing biohydrogen and carboxylic acids production from brewery spent grains: Microbial dynamics and biochemical analysis" was published in 2022. Journal: Eng Life Sci.

## 3 RESULTS AND DISCUSSION

### 3.1 Metals addition improves carboxylic acids (CA) output

The reactor operated with an inoculum supplemented with iron exhibited the highest CA production (R_Fe_: 29.13 gCOD/L), followed by reactors supplemented with cobalt (R_Co_: 28.87 gCOD/L), zinc (R_Zn_: 24.74 gCOD/L), and nickel (R_Ni_: 23.77 gCOD/L) (Figure 1A). These values were 1.74, 1.72, 1.47, and 1.42 times higher than the control (R_CTRL_: 16.72 gCOD/L), respectively. Solvents, such as ethanol and butanol were also produced in the reactors at varied concentrations. When all metals were combined, the production of CA was 2.6 times higher than in the control and corresponded to a yield of 0.44 g/gVS. In comparison, the yield from the other reactors was 0.29 g/gVS (R_Fe_) > 0.28 g/gVS (R_Co_) > 0.24 g/gVS (R_Zn_) > 0.23 g/gVS (R_Ni_) > 0.16 g/gVS (R_CTRL_) (Figure 1B).

**FIGURE 1:** (A) Metabolites production from acidogenic fermentation of BSG (B) yields of CA accumulated by the end of the experiment (day 72)

### 3.2 Metal shock alters the composition of CA

Total CA included SCCA, such as acetic, propionic, isobutyric, butyric, isovaleric, and valeric acids, as well as MCCA such as caproic acid (Figure 2A–F). Compared to the control reactor, metal supplementation selectively enhanced acetic and butyric acid biosynthesis. Production of individual CA increased gradually up to a certain point and stabilized thereafter. The subsequent decline of some of them indicated their conversion to MCCA. The highest acetic acid production was 5.13 gCOD/L (R_Co_), followed by 4.8 gCOD/L (R_Fe_), 4.14 gCOD/L (R_Zn_), and 3.95 gCOD/L (R_Ni_); whereas R_CTRL_ generated only 2.68 gCOD/L of acetate. Butyric acid biosynthesis became dominant in the reactor dosed with iron (11.4 gCOD/L), followed by R_Zn_ (8.9 gCOD/L), R_Ni_ (8.52 gCOD/L), R_Co_ (7.94 gCOD/L), and R_CTRL_ (7.61 gCOD/L). Together, acetic, and butyric acid amounted to 55.74%, 52.77%, 50.51%, 45.16%, and 67.66% of overall CA content, respectively. Propionic acid biosynthesis was greater in R_Fe_ (0.42 gCOD/L) among metal‐dosed reactors (the others reached 0.33–0.35 gCOD/L), but still lower than in R_CTRL_ (1.77 gCOD/L). Higher production of valeric acid was noticed in R_Fe_ (3.75 gCOD/L); whereas isovaleric acid was higher in R_Co_ (1.63 gCOD/L) and R_Zn_ (1.22 gCOD/L). Ethanol production was as follows: R_Co_ (3.29 gCOD/L) > R_Zn_ (1.79 gCOD/L) > R_Ni_ (0.79 gCOD/L) > R_Fe_ (0.77 gCOD/L) > R_CTRL_ (0.64 gCOD/L). However, ethanol content decreased with time, indicating its progressive consumption. Butanol production was observed only in reactors dosed with metals: R_Zn_ (2.90 gCOD/L) > R_Co_ (1.17 gCOD/L) > R_Fe_ (0.88 gCOD/L) > R_Ni_ (0.80 gCOD/L).

The article "Effect of metals on the regulation of acidogenic metabolism enhancing biohydrogen and carboxylic acids production from brewery spent grains: Microbial dynamics and biochemical analysis" was published in 2022. Journal: Eng Life Sci.

**FIGURE 2:** Change in microbial metabolites with respect to different metals addition

### 3.3 Metals exert a synergistic effect on acidogenic metabolites

The combination of all four metals and its influence on acidogenic metabolites was evaluated with respect to SCCA and MCCA production. Overall production of CA reached 45.84 gCOD/L in R_MIX_, corresponding to 3.02 times more than in the control reactor (Figure 2F). Almost 49.66% of this amount was contributed by acetic and butyric acid, with 9.03 gCOD/L and 12.59 gCOD/L, respectively. Propionic acid contributed with 4.29 gCOD/L, which was 2.43 times more than in the control reactor and 13.52, 12.91, 12.35, and 10.14 times more than the individual effects of nickel, cobalt, zinc, and iron, respectively. This striking production of propionic acid points to the stimulatory effect of the metal mixture. Other metabolites that displayed a significant increase were isobutyric (1.82 gCOD/L), isovaleric (0.8 gCOD/L), and valeric (4.28 gCOD/L) acids, whose amounts were 6.25, 1.56, and 2.5 times greater than in R_CTRL_. By the end of the experiment, MCCA accumulation reached 10.17 gCOD/L, which was 4.71 times higher than in R_CTRL_ and 1.31, 1.13, 0.95, and 0.85 times higher than with individual supplementation of iron, zinc, nickel, and cobalt, respectively. The combination of metals in the reactor further increased the proportion of acetate (7.4 gCOD/L) and butyrate (15.36 gCOD/L), which represented 51.6% of total CA. As a result of increased acidogenesis, the higher NADH/NAD^+^ ratio had to be balanced by activation of the propionic acid pathway, with consequent generation of more NAD^+^ [20]. Therefore, the synergistic effect of the various metals manifested as improved solvents production. Specifically, the mixture of zinc and cobalt enhanced propionic acid, as well as ethanol and butanol output, confirming a previous observation by Dahiya et al. (2020) on ethanol and propionic acid biosynthesis [11]. In particular, Dahiya et al. [11] reported the synergistic effect of zinc and cobalt on ethanol production comparing two metals being added separately.

The article "Effect of metals on the regulation of acidogenic metabolism enhancing biohydrogen and carboxylic acids production from brewery spent grains: Microbial dynamics and biochemical analysis" was published in 2022. Journal: Eng Life Sci.

### 3.4 MCCA production without an external electron donor

Formation of MCCA requires an electron donor in the form of ethanol, methanol, lactic acid or butanol [3, 21, 22]. In this respect, chain elongation of protein‐based substrates remains poorly explored. Amino acids within proteins can act as both electron acceptors and donors, and can efficiently undergo chain elongation during the fermentation process without the need for external electron donors [23, 24]. Our previous study on BSG as substrate revealed protein‐based chain elongation without addition of any electron donor during production of 8.95 gCOD/L MCCA [24]. Figure 2 summarizes the MCCA production pattern from reactors operated for 72 days. Up until day 12, MCCA production was minimal in all reactors (0.45–1.29 gCOD/L) and represented only 13%–28% of the total CA accumulation. Production gradually increased in all reactors and by day 24, it amounted to 6.22 gCOD/L with R_Co_, but remained below 5 gCOD/L with all other rectors. MCCA production peaked by day 60 and stabilized thereafter. The concentration of caproic acid was enhanced mainly in R_Co_ (12.03 gCOD/L), achieving a 5.57 times higher titer than R_CTRL_ (2.16 gCOD/L). The concentrations of caproic acid recorded with the other metals were 10.71 gCOD/L (R_Ni_), 9.03 gCOD/L (R_Zn_), and 5.8 gCOD/L (R_Fe_), which corresponded to 4.97, 4.1, and 3.5 times more than the control and represented 36%–45% of the net CA accumulation.

### 3.5 Addition of metals promotes biohydrogen production

Figure 3 shows the influence of metals on bioH_2_ production. BioH_2_ is generated together with CA through the acetic and butyric acid pathways (Equations 1 and 2).

(1) $$\begin{array}{c} C_{6}H_{12}O_{6}+2H_{2}O\to 2CH_{3}\mathrm{COOH}+2CO_{2}+4H_{2} \end{array}$$

(2) $$C_{6}H_{12}O_{6}\to CH_{3}CH_{2}CH_{2}\mathrm{COOH}+2CO_{2}+2H_{2}$$

**FIGURE 3:** (A) Cumulative biohydrogen production (B) biohydrogen yield recorded from different bioreactors

Most bioH_2_ was produced during the initial phase of the operation (until day 12), diminishing thereafter (Figure 4A). In fact, 70%–80% of volumetric bioH_2_ production was documented within the first 3 days of fermentation in all reactors: R_Fe_ (5.28 L; 82.4%) > R_Co_ (4.6 L; 82.9%) > (3.48 L; 75.9%) > (2.38 L; 84.3%) > (2.1 L; 78.6%). From day 4 until day 12, an additional 1.12 L were accumulated in R_Fe_, 1.1 L in R_Ni_, 0.96 L in R_Co_, 0.57 L in R_CTRL_, and 0.44 L in R_Zn_, amounting to an overall production of 6.4 L, 4.59 L, 5.65 L, 2.67 L, and 2.82 L, respectively. Elevated bioH_2_ production in R_Fe_ can be attributed to the involvement of iron in hydrogenase activity, substrate utilization, and a general stimulatory effect on microorganisms. Hydrogenases catalyze the efficient conversion between H^+^, electrons, and H_2_. The [Fe–Fe] hydrogenase is the most effective at reducing H^+^ to molecular H_2_ [25]. Indeed, the addition of metals/nanoparticles has been widely applied to enhance hydrogenase activity in various metabolic pathways using different organic substrates. Lee et al. [26] reported a bioH_2_ production rate of 24 ml/gVS/h and maximum yield of 0.8 g/L (131.9 ml/g_sucrose_) upon addition of 4 g/L FeCl_2_. Whereas iron addition favors bioH_2_ production, its limitation has been shown to decrease hydrogenase activity, with solvent production replacing acidogenesis [27]. In this study, the addition of metals promoted bioH_2_‐producing pathways, as indicated by increases of 157.9% (R_Fe_), 127.12% (R_Co_), 126.82% (R_Zn_), and 116.74% (R_Ni_) in acetic and butyric acid output compared to R_CTRL_. Concomitantly, these metals promoted low propionic acid production, whose biosynthesis pathway does not generate bioH_2_.

The article "Effect of metals on the regulation of acidogenic metabolism enhancing biohydrogen and carboxylic acids production from brewery spent grains: Microbial dynamics and biochemical analysis" was published in 2022. Journal: Eng Life Sci.

**FIGURE 4:** (A) Ammonium production, (B) dehydrogenase activity recorded with respect to fermentation time

The resistance or acclimatization to bioH_2_ production might differ between reactors owing to shifts in metabolic pathways caused by different metals. Zhang et al. attained a 15% higher bioH_2_ yield with 8% enhanced acetic acid production [20]. In this study, the lower bioH_2_ evolution observed in the control reactor might be explained by its 4–5.5 times higher propionic acid production compared to metal‐supplemented reactors. BioH_2_ output in R_MIX_ was initially higher than in other reactors, with almost 90% (4.62 L) of total volumetric bioH_2_ observed within day 3, and only 0.47 L observed between day 4 and day 10 (cumulative: 5.09 L). As discussed in Section 3.4, the enhanced acidogenic activity in R_MIX_ had a positive effect on bioH_2_ output. Similarly, Gadhe et al. obtained more bioH_2_ by adding nanoparticles containing both Fe_3_O_4_ and NiO than with nanoparticles bearing only one metal compound [7]. This can be explained by combinations of different metal‐containing nanoparticles promoting electrical conductivity and thus accelerating the transfer of electrons to the hydrogenase active site during bioH_2_ production [28]. Ferredoxin is an important redox mediator, assisting the conversion of pyruvate to acetic acid and CO_2_ [29]. Here, the reactor supplemented with iron attained the highest yield (91.56 ml H_2_/gVS load), followed by R_Co_ (80.77 ml H_2_/gVS load), R_MIX_ (72.74 ml H_2_/gVS load), R_Ni_ (65.63 ml H_2_/gVS load), R_Zn_ (40.32 ml H_2_/gVS load), and R_CTRL_ (38.19 ml H_2_/gVS load) (Figure 3B). While the bioH_2_ potential of R_MIX_ was slightly lower compared to R_Fe_ and R_Co_, this was compensated by its much higher acidogenic and acetogenic potential, and exemplified the synergistic role of metals in microbial metabolism. Zinc plays various roles in H_2_ production [30]. On the other side, a good bioH_2_ yield in R_Ni_ might derive from participation of Ni as a co‐factor in [Fe‐Ni] hydrogenases, which reduce protons using electrons transferred by [Fe–S] clusters [25]. [Ni–Fe] hydrogenases are the most common in nature, but [Fe–Fe] hydrogenases are the most active in terms of H^+^ reduction and H_2_ output. An increasing the concentration of metals has a positive effect on volumetric bioH_2_ output; excessive metal loads may decrease production due to increased toxicity. Such phenomenon was not observed in this study, which might be explained by acclimatization of the microbes to the environment. Although bioH_2_ production decreased gradually after day 9, the continuous production of CA until day 60 indicated the persistent microbial conversion of substrate.

### 3.6 Ammonium production

Microbial ammonium production from proteins and their derivatives occurs via many processes, such as proteolysis, peptide degradation, deamination, and deamidation [31]. Moreover, an environment rich in H_2_ provides an opportunity for direct production of ammonia following reaction with nitrogen [32]. As shown in Figure 4A, the highest amount of ammonium was attained in R_Fe_ (0.36 mol), followed by R_Co_ (0.31 mol) and R_Zn_ (0.25 mol); whereas R_Ni_ (0.16 mol) was similar to R_CTRL_ (0.17 mol) (Figure 4A). In comparison, the mixture of metals yielded 0.34 mol, equivalent to 2.00, 1.84, 1.33, and 1.11 times more ammonium than R_CTRL_, R_Ni_, R_Zn_, and R_Co_, respectively, but still not as much as R_Fe_. Ammonia controls the redox balance in the reactor, particularly when the acidogenic pathway proceeds to methanogenesis and the accumulated CA are transformed to methane; under these circumstances, ammonia ensures medium alkalinization. In this study, the bioprocess was designed to favor the accumulation of CA and prevent their conversion to methane. Consequently, the pH shifted gradually from pH 7 to acidic (pH 4.9–6.1), without any further alterations. Additionally, ammonium contributes to in situ buffering by neutralizing the CA present in the reactor. In this study, a higher ammonium output upon metal supplementation neutralized more CA and stabilized the pH of the reactors, further promoting acidogenic fermentation. Ammonium is the precursor for ammonia; hence, its release from waste/wastewater adds value to the whole process [33].

The article "Effect of metals on the regulation of acidogenic metabolism enhancing biohydrogen and carboxylic acids production from brewery spent grains: Microbial dynamics and biochemical analysis" was published in 2022. Journal: Eng Life Sci.

### 3.7 Dehydrogenase activity

Different dehydrogenases are required for the oxidation and reduction of organic compounds. Here, the electron acceptors were assessed based on the reduction of TTC to triphenyl formazan. Transfer of H^+^ between metabolic intermediates through redox reactions is catalyzed by dehydrogenases using several cofactors, such as NAD^+^ and FAD^+^. Dehydrogenase activity was relatively high between day 12 and day 24, but decreased gradually thereafter (Figure 4B), correlating well with the production of acidogenic metabolites in all reactors (R^2^ = 0.91–0.97). The proportion of CA generated during this process is the key indicator of H_2_ output. The mixture of metals favored dehydrogenase activity (22.8 μg/ml), which surpassed those achieved in R_Fe_ (19.2 μg/ml), R_Zn_ (17.3 μg/ml), R_Co_ (16.8 μg/ml), R_Ni_ (14.2 μg/ml), and R_CTRL_ (13.4 μg/ml). Starting on day 24, dehydrogenase activity manifested first a slight and then a more sustained decline, falling to 8.5–13.1 μg/ml by day 36 (4.9 μg/ml in R_CTRL_), and then to between 2.33 and 0.12 μg/ml from day 48 onward. The obtained results reflect the active role of oxidoreductases, as well as the efficiency with which microorganisms adapted to the selective pressure imposed by a metal‐rich environment.

### 3.8 Addition of metals causes a shift in functional microbial communities

As shown in Figure 5A, microbial community composition exerted a strong influence on the production of CA and bioH_2_ from BSG in a metal‐rich environment. Despite a high metal concentration, stable growth and propagation of microorganisms demonstrated the strong adaptability and functional capacity of microorganisms present in the reactors. At the phylum level, the predominant taxa were Firmicutes, Bacteroidota, Actinobacteriota, Chloroflexi, Halobacterota, Proteobacteria, Caldatribacteriota, and Desulfobacterota (Figure 5A). These taxa are common in anaerobic digesters, whereby they degrade organic matter into bioH_2_ and CA [34]. In particular, Firmicutes increased from 33.42% (R_CTRL_) to 90.3% in R_Co_, 84.51% in R_Fe_, 83.7% in R_Ni_, and 64.93% in R_Zn_. This increment can be attributed mainly to enrichment with the class Clostridia in all metal‐supplemented reactors, where they accounted for 78.82% (R_Fe_), 77.58% (R_Co_), 75.81% (R_Ni_), and 58.86% (R_Zn_) of genera, but only 20.94% in the control. Interestingly, the percentage of Firmicutes was even higher (93.06%) when the metals were combined, further confirming a synergistic action of metals during fermentation. Another dominant phylum was *Bacteroidota*, although its abundance varied greatly between reactors, from 41.25% in R_CTRL_ to 23.16% in R_Zn_, 11.82% in R_Fe_, 8.34% in R_Co_, and 4.51% in R_MIX_. The abundance of the 30 most common genera in the different reactors is depicted as a heatmap in Figure 5B. The microbial culture in the control reactor (R_CTRL_) was the most dissimilar compared to all other reactors, suggesting a significant shift in microbial community composition in response to metal addition. None of the reactors shared the same pattern, which could be ascribed to the role of individual metals in the fermentation process. The addition of cobalt led to the dominance of *Enterococcus* (13.27%), *Clostridium sensu stricto 1* (10.82%), *Caproiciproducens* (10.68%), *Clostridium sensu stricto 12* (8.24%), *Lacticaseibacillus* (6.71%), *Romboutsia* (6.58%), *Paraclostridium* (5.14%), and *Prevotella* (4.50%). Instead, the addition of iron favored the proliferation of *Clostridium sensu stricto 1* (54.47%), *Prevotella* (11.63%), *Caproiciproducens* (4.95%), *Romboutsia* (3.67%), *Clostridium sensu stricto 18* (2.57%), *Megasphaera* (2.23%), and *Bacillus* (2.02%). These changes in bacterial community composition indicated that bioH_2_ and CA producers, particularly the chain‐elongating bacteria, became more competitive and contributed to increased production of caproic acid. The relative abundance of bioH_2_ and acid‐producing bacteria such as *Clostridium sensu stricto 1* in R_Fe_ may explain the strong accumulation of CA in this reactor. The dominance of this genus was as follows: 54.47% (R_Fe_) > 34.44% (R_Co_) > 31.84% (R_Ni_) > 27.74% (R_Zn_) > 9.74% (R_MIX_) > 5.13% (R_CTRL_). *Clostridium sensu stricto 1* is known for effective bioH_2_ production from multiple feedstocks, including food waste, lignocellulosic biomass, sucrose, starch, hemicellulose, glucose, cellulose, and sewage sludge [35, 36]

**FIGURE 5:** (A) Microbial community structure in each sample, (B) heat map of genera level community composition observed in different reactors comparing with control

The production of MCCA in the reactors can be linked to the genus *Megasphaera* as many of its members such as *Megasphaera elsdenii* are capable of chain elongation from glucose and lactic acid [22]. An enhanced production of acetic acid in this study particularly with R_MIX_ can be attributed to the association and synergy between metals, resulting in the dominance of *Clostridium sensu stricto* *5* species, which are homoacetogens and convert C1 compounds to acetic acid (4H_2_ + 2CO_2_ → CH_3_COOH + 2H_2_O), along with other acid producers, such as *Clostridium sensu stricto 1*, *Clostridium sensu stricto 12*, and *Clostridium sensu stricto 18*. Accordingly, the mixed metal strategy can favor a biocatalyst that regulates the process by stimulating the proliferation of specific microorganisms and production of specific metabolites. Besides bioH_2_ producers, the obligate anaerobes *Paraclostridium* (R_Fe_ and R_Zn_) and *Terrisporobacter* (0.32%–1.51%) were also detected in the reactors. *Paraclostridium* can use a variety of organic carbon sources for its growth; with some species of this genus effectively hydrolyzing starch [37]. The acetic acid producer *Terrisporobacter* has the capability to form endospores under harsh conditions [38]. Notably, the bioH_2_‐producing genus *Enterococcus* was enriched in R_Co_. The Ruminococcaceae family in the Firmicutes phylum was represented exclusively by the genus Ruminococcus, comprising fibrolytic bacteria that hydrolyze polysaccharides and ferment hexoses and pentoses to produce bioH_2_. The same genus has been reported to generate acetic and propionic acid under different pH conditions [39, 40]. Production of butyric and valeric acid by some genera of the *Ruminococcaceae* has been reported [41]. Under acidic pH, the *Ruminococcaceae* strain CPB6 was found to generate caproic acid [42]. In this study, the proliferation of *Ruminococcaceae* was favored in R_MIX_ (21.32%) compared to supplementation with single metals (4.75% in R_Co_, 2.86% in R_Ni_, 1.22% in R_Fe_, and 0.94% in R_Zn_) or R_CTRL_, whereby it was not detected. Another genus, which dominated the metal‐rich reactors was Romboutsia, which is known for the fermentation of glucose into acetic, isobutyric, and isovaleric acids. Romboutsia was predominant under cobalt supplementation: 22.1% (R_Co_) > 16.28% (R_Ni_) > 14.18% (R_Zn_) > 12.61% (R_MIX_) > 4.56% (R_CTRL_) > 3.67% (R_Fe_). Most bioH_2_ production in R_CTRL_ can be attributed to an abundance of *Prevotella* species, which assimilate soluble sugars to bioH_2_ [43]. *Clostridium* species are very effective bioH_2_ producers that use carbohydrates as substrate. Instead, amino acids derived from protein degradation cannot be easily used for bioH_2_ production because of their unique molecular structure and low C/N ratio. Rather, amino acids can be anaerobically degraded to CA by a mixed culture of *Clostridium* species in a coupled oxidation‐reduction reaction. The dominance and function of microorganisms in the metal‐rich reactors was dictated by their physiological activity and mutual interaction.

The article "Effect of metals on the regulation of acidogenic metabolism enhancing biohydrogen and carboxylic acids production from brewery spent grains: Microbial dynamics and biochemical analysis" was published in 2022. Journal: Eng Life Sci.

## 4 CONCLUSION

This study documented the influence of elevated concentrations of metals on acidogenic fermentation. Production of CA was significantly enhanced in response to metal addition, leading to yields of 0.27–0.33 gCOD/gVS, which were much higher than in the control reactor (0.17 gCOD/gVS). A similar improvement was observed for bioH_2_ production, particularly with iron, which can be attributed to the coordinating role of this metal within hydrogenases. Furthermore, changes in bacterial diversity and richness of *Firmicutes* indicated good adaptation of the microbial community to pressure arising from a metal‐rich environment, and exemplified by an increment in dehydrogenase activity. Metal supplementation in a combined or individual form represents a promising strategy for regulating the bioprocesses that control the generation of numerous commercially interesting acidogenic metabolites from renewable feedstocks.

## CONFLICT OF INTEREST

The authors declare that they have no known competing financial interests or personal relationships that could have appeared to influence the work reported in this paper.

## Data Availability

The data that support the findings of this study are available from the corresponding author upon reasonable request.
